# COVID-19 Epidemic Analysis in India with Multi-Source State-Level Datasets

**DOI:** 10.1155/2022/2601149

**Published:** 2022-04-25

**Authors:** Qirui Wang

**Affiliations:** Fok Ying Tung Graduate School, The Hong Kong University of Science and Technology, Hong Kong 999077, China

## Abstract

The COVID-19 pandemic has been a global crisis affecting billions of people and causing countless economic losses. Different approaches have been proposed for combating this crisis, including both medical measures and technical innovations, e.g., artificial intelligence technologies to diagnose and predict COVID-19 cases. While there is much attention being paid to the USA and China, little research attention has been drawn to less developed countries, e.g., India. In this study, I conduct an analysis of the COVID-19 epidemic in India, with datasets collected from different sources. Several machine learning models have been built to predict the COVID-19 spread, with different combinations of input features, in which the Transformer is proven as the most precise one. I also find that the Facebook mobility dataset is the most useful for predicting the number of confirmed cases. However, I find that the datasets from different sources are not very effective when predicting the number of deaths caused by the COVID-19 infection.

## 1. Introduction

Reoccurring outbreaks of the COVID-19 epidemic in the world remind us that the coronavirus is becoming more dreadful. Especially the various variants, which are threatening the current protection systems and affecting the reliability of vaccination. Among various variants, Delta and Delta-plus, which were first discovered and initially spread in India, showed breathtaking infectivity. On May 5, over 400 thousand people have been confirmed in a day in India.

Compared with other countries, the consistency of coronavirus in India is purer, and the related studies have a higher value as the reference for Indian and other governments preventing the Delta and Delta-plus variant. This is a merit chance to disclose more information about the new variants, including whether the current government's controlling methods still work, could the mobility data still be helpful for predicting the trend of epidemic, or determine the effect of Indian vaccination for the new situation. However, there is little research on the Indian epidemic and rarely adopts complex and state-of-art machine learning models. One of the reasons for the situation is insufficient public or complete Indian epidemic datasets. Some related institute in India does not public the historical data but daily data, and it will be time-costing to collect data by researchers. The missing values in the collection of the epidemic datasets also disturb the researches. Also, the short of attention of the Indian epidemic is also a problem.

In this research, I mainly did the following contributions: (I) Collecting an Indian with the statewise COVID-19 dataset covering from October 1, 2020, to July 15, 2021, with medical statistics, population mobility, and census data. Considering the complex situation of Indian society and geography, a statewise dataset will be beneficial for evaluating the importance of features and show the influences at the geography level. The dimensions of my dataset are much more than previous, and the dataset will be public on GitHub (the website of data: http://github.com/vividricky/IndiaCovid19StateDataset) and convenient for the following researchers. (II) Six different models have been implemented and compared in the research, including traditional statistic models, logistic regression, and multiple linear regression, the data-driven time-series machine learning models: LSTM, Transformer, DeepAR, and TCN for predicting the trend of COVID-19 in India. Specified notes that up to the research finished, few studies have tried the last three models in the Indian epidemic. This work fills the gap of state-of-art time-series machine learning in this field. According to the experiment, the Transformer model showed the best performance during six models, and mobility data contributes most in predicting the trend of the epidemic.

Based on my observations, I demonstrate that the collection of multisource datasets is valuable for the prediction and further control of the COVID-19 epidemic, although its cost is a new burden for the government. The second corollary is that human mobility does contribute significantly to the spread of viruses, including COVID-19 and other influenza and diseases. Maintaining social distance and lockdown policies are necessary even with the potential economic losses.

The rest of this paper is organized as follows. Related work is discussed in Section 2. Multi-source datasets are described in Section 3. The models used in this study are discussed in Section 4. The experimental results are presented in Section 5. A short conclusion is given in Section 6.

## 2. Related Work

Since the first break out of the COVID-19 epidemic in India, many researchers have contributed to identifying factors that may influence the spread of COVID-19 and constructing models to predict the number of confirmations, deaths, and recoveries in India. These models cover medical, mathematical, and machine learning types. Also, some studies for other countries provide a good reference for studying the situation in India.

Mele and Magazzino investigated the relationship between economic growth, air pollution, and transmission of COVID-19 in India [1]. They first used stationarity and Toda-Yamamoto causality to prove that PM2.5, CO2, and NO2 increase with the development of cities. Then, a D2C algorithm is adopted to verify a casual line between PM2.5 and the number of deaths of COVID-19. Roy et. al did the disease risk analysis of Indian states [2]. They forecast the risk of COVID-19 using Autoregressive Integrated Moving Average (ARIMA). They introduce the GIS data of India into the model, including the population density and regional status. ARIMA captures the pattern in two parts, in which AR calculates based on the past values and MA computes the difference of current and previous knowledge. However, ARIMA only considered the time-dependent data and cannot understand the breaking events, such as community infections. Kumari et al. built a multiple linear regression model of social policies to predict the spread, recovery, and deaths in India [3]. Multiple linear regression is an explained method that can tell the importance of factors by showing weights. Moreover, autoregression and autocorrelation have been imported to the model to increase the accuracy of the model and finally generate a good performance. As shown in the research of [3], the lockdown and social distance policies contribute the most to slow the spread of the virus.

Besides the traditional mathematic models, medicinal models and machine learning models are also widely used in related studies. Ghosh and Malavika's teams successively used the logistics regression model to predict the trend of COVID-19 [4, 5]. Ghosh et al. separately developed a logistic regression model and an exponential regression model [4]. They used the exponential regression model as the upper bound and a linear combination model of the above two models with DIR value as the lower bound to predict the range of confirmed numbers in India. Foy et al. focused on the priority group of vaccination. They considered the age structure and implemented the SEIR model to simulate [6]. As the result, the elder, who are the most vulnerable to COVID-19, should be inoculated immediately. Malavika et al. used a modified logistic growth model, which involved the population of the region to predict the number of confirmed, achieving a good performance. Shrivastav and Jha discussed the impact of temperature and humidity on the transmission of COVID-19 [7]. They constructed a gradient boosting model (GBM) with maximum and minimum temperature and humidity data of Indian states to forecast. In addition, they also provided ANOVA analysis of atmospheric data and COVID-19 data. Chandra et al. implemented the LSTM models to predict the trend based on the time-series data [8]. According to experiments, LSTM had a better performance than ED-LSTM and BD-LSTM with limited data, and the authors also believed that the model can be improved by introducing more data. Moreover, their work also shows the possibility for the long-term prediction of Indian epidemic situation.

According to related studies, on the one hand, the prediction of the spread of the COVID-19 is a complex task involving multiple aspects of society. Based on this understanding, introducing more features in the model may contribute to the accuracy and stability of the model [1–3, 6, 7]. In my study, more medical, population density, and population mobility data were collected for the model, which are more direct to the spread of the virus. These characteristics were introduced for the first time in the COVID-19 outbreak in India before the study was completed. On the other hand, the previous researches have proved the feasibility of their selecting models but have their own limitations. Traditional mathematical models are interpretable, but lack the ability to effectively predict epidemic trends [1–3]. The time-series deep learning models describe the spread of COVID-19 [8] better than regression models [3–5]. However, there are few studies addressing related research. In this study, a more advanced time-series deep learning model will be implemented to fill the gap of these studies for the Indian epidemic. Moreover, previous researchers have collected data only for some cities or the whole country. It did not take into account the complexities of Indian society, and with the advancement, my study does experiments at the national level.

## 3. Data Collection and Processing

### 3.1. Raw Data Sources

This study analyzed and constructed models using multiple sources, including medical statistics, population mobility, and census data under COVID-19. Considering the reliability of the data sources, the datasets selected for this study meet at least one requirement: (1) data collected and published by official agencies (MoHFW Vaccines and Indian Census 2011) and (2) research datasets that are widely cited in academic papers (COVID-19 India, Google mobility, and Facebook mobility).

The medical statistics consist of two datasets. As shown in Figure 1, the COVID-19 India dataset records the number of confirmations, recoveries, and deaths per state per day, with each state abbreviated, e.g., ap a for Andhra Pradesh. As shown in Figure 2, the Ministry of Health and Family Welfare vaccination data is derived from the daily data published by the Ministry of Health and Family Welfare (MoHFW), Government of India. It contains the cumulative number of vaccinated beneficiaries, including first, second, and total doses. Special note, data became available on February 24.

Population mobility data includes Google mobility and Facebook mobility data. Google community mobility collects trends in population mobility in parks, workplaces, bus stops, retail, entertainment, grocery stores, pharmacies, and residences. Meanwhile, the Facebook Data for Good project quantifies mobility trends and residency values in the area.

The Indian census 2011 dataset (Data source website: http://www.census2011.co.in/district.php) contains the related information of India census 2011 which will be used to calculate the immune rate and state-level mobility in 3.2 part.

The range of dates is mainly covering from October 1, 2020, to July 15, 2021, and the time period is day. All data are collected from available public sources.

The raw data sources are shown in Table 1.

Please note that the website of MoHFW does not record the historical data. The daily data need to be crawled by the user. The crawled data in this study will also be shared in the GitHub later.

The raw dataset description is given in Table 2.

### 3.2. Data Preprocessing

Standardization and merging of datasets is challenging due to the diverse data sources and complex social conditions in India. Finally, the following issues were addressed in the pre-processing process: (i) standardized the storage format as CSV. For the MoHFW Vaccination data, I imported the Tabula package to convert the data from PDF to CSV format. Also, I added a step to verify the correction of converting by checking the equality of the sum of the first dose number and second dose number to the total dose number. (ii) Second is the standardized the state names through different data sources. (iii) Third is the standardized the district names. Special notes that some districts in India do not have a sole office spell. My dataset has standardized the district names by referring to the office Indian directory website (http://www.goidirectory.gov.in/). (iv) Fourth is by adding the new districts created after the 2011 to Indian census 2011 dataset, the population numbers were estimated based on original regions. The whole workflow of preprocessing can refer in Figure 3.

In the state-level Facebook mobility, since the target dataset is focused on the state level but Facebook mobility records the data at the district level, we need to aggregate these data for further handling. In this case, the district contributes mobility values based on the ratio of the district's population to the state's population. The state population is calculated based on the grouping of districts in the India 2011 Census dataset. This is shown in the following equation:

(1) $$\begin{array}{c} \text{S}=\underset{\text{i}=1}{\sum }\alpha_{\text{i}}{\text{M}}_{\text{i}}, \end{array}$$

where *S* represents the State's mobility and *M*_*i*_ and *α*_*i*_ separately represent the *i*th district's mobility and ratio population of the state.

In handing the missing value, the dataset contains two types of missing values. (1) Part of the features cannot cover the whole-time range which is vaccination data in this case. Considering the limited ratio of beneficiaries vaccinated in the starting. I used 0 to fill these missing values. (2) Some missing values are generated by statistical work and data collection. For the gaps which are small, the data would be filled with the previous time step data to fulfill the missing value. For the gaps which are obvious, the current districts or states' data will be dropped.

### 3.3. Data Description

The final dataset holds data for each of the 33 states or union territories, covering the dates from October 1, 2020, to June 30, 2021. The four union territories of Andaman and Nicobar Islands, Dardala and Nagar Haveli, and Ladakh and Lakshadweep have huge gaps in data collection and will not be used for model construction. Although Telangana has been separated from Andhra Pradesh, these two states will be recorded together in order to minimize errors in manual division of data.

Each state data has 273 rows with 14 columns. The detailed information of features is explained in Table 3.

### 3.4. Shortage of Dataset

Except four union territories data has not been recorded, the population of some districts created after 2011 may also been calculated repeated. These new districts' population are estimated based on the original region's population that are statistic in 2011, and these regions may belong to different districts before they are independent. It may lead to double counting in the sum of population. Meanwhile, the Telangana also covers some region past belong to other state but not only Andhra Pradesh. However, the sum of these potentially confounding population is smaller than the three percent of the country population, which can generate limited effect to the model.

## 4. Methodology

The research of [8] showed the feasibility of time-series deep learning models in predicting the Indian epidemic. In this section, I will present different models used to predict the number of confirmed cases and deaths of COVID-19. These models were chosen because they have been shown to be effective in a range of problems in different domains [11–13]. I wanted to validate their performance in the new crown outbreak prediction task.

### 4.1. Logistic Regression

The logistic regression model [14] is popular in relevant studies, as it is capable of capturing the effect of the government's preventive measures [4] and it is believed that logistics regression follows the trend of Coronavirus outbreak [5].

The logistic regression model is formulated as follows:

(2) $$\begin{array}{c} \text{y}=\frac{1}{1+{\text{e}}^{-{\text{w}}^{\text{T}}\text{x}}}, \end{array}$$

where *y* is the prediction number of current state's confirmed cases, *x* is the current input, and w is the model parameter.

### 4.2. Multiple Linear Regression

Multiple linear regression [14] is a basic and popular statistic model. It only requires minimum computing resources to construct the model and can be explained by comparing the weights of parameters.

The multiple linear regression model can be stated as follows:

(3) $$\begin{array}{c} \text{y}={\text{b}}_{0}+{\text{b}}_{1}{\text{x}}_{1}+{\text{b}}_{2}{\text{x}}_{2}\cdots {\text{b}}_{\text{n}}{\text{x}}_{\text{n}}, \end{array}$$

where *b*_*i*_ is the weight of current input item *x*_*i*_ and is estimated by the least squares method.

### 4.3. Long Short Term Memory (LSTM)

Compared with both traditional time-series models and standard recurrent neural networks (RNNs), long short term memory (LSTM) [15] shows a better performance in handling the long-term dependency relationship by using the LSTM cell shown in Figure 4.

Figure 4 shows the structure of a LSTM cell, which would be noted as *L* in Figure 5. Three red dotted bordered boxes represent three different gates in LSTM, namely, forget gate, input gate, and output gate from left to right. The forget gate controls the keeping or throwing of input information from the cell state as follows:

(4) $$\begin{array}{c} {\text{f}}_{\text{t}}=\sigma \left({\text{W}}_{\text{f}}{\text{x}}_{\text{t}}+{\text{U}}_{\text{f}}{\text{h}}_{\text{t}-1}+{\text{b}}_{\text{f}}\right), \end{array}$$

where *x*_*t*_ denotes the input features and *h*_*t*_ denotes the hidden states. *W* ∈ *R*^*h*×*d*^ and *U* ∈ *R*^*h*×*h*^  are weight parameter matrices, and *b* ∈ *R*^*h*^ is the basis parameter vector.

The input gate decides which values will be updated in the cell states and be denoted as follows:

(5) $$\begin{array}{c} {\text{I}}_{\text{t}}=\sigma \left({\text{W}}_{\text{i}}{\text{x}}_{\text{t}}+{\text{U}}_{\text{i}}{\text{h}}_{\text{t}-1}+{\text{b}}_{\text{i}}\right),\\ {\bar{C}}_{t}=\tan h\left(W_{C}x_{t}+U_{C}h_{t-1}+b_{C}\right),\\ {\text{C}}_{\text{t}}={\text{f}}_{\text{t}}○{\text{C}}_{\text{t}-1}+{\text{I}}_{\text{t}}○{\bar{\text{C}}}_{\text{t}}, \end{array}$$

where ${\bar{C}}_{t}$ restores the candidate values which may be added into cell states and  *C*_*t*_ represents the internal memory of a LSTM unit.

The output gate controls the output of the cell states as follows:

(6) $$\begin{array}{c} {\text{O}}_{\text{t}}=\sigma \left({\text{W}}_{\text{o}}{\text{x}}_{\text{t}}+{\text{U}}_{\text{o}}{\text{h}}_{\text{t}-1}+{\text{b}}_{\text{o}}\right),\\ h_{t}=O_{t}*\tan h\left(C_{t}\right). \end{array}$$

### 4.4. Transformer

The mission of Transformer [16] is to decide what parts of input should be focused on by introducing the attention mechanism. Another important feature of the Transformer is the encoder-decoder structure. Different from traditional time-series models, which encode the input one-time step at a time, the Transformer encodes all the input simultaneously.

The architecture of the Transformer is shown in Figure 6. The left part represents the encoder block, and the right part represents the decoder block. After the embedding operation is completed, the inputs are fed to the self-attentive layer. In the self-attentive case, each input has three matrix vectors Q, K, and V, representing query, key, and value, respectively. First, these matrices are used for scaled dot product attention with the following equation:

(7) $$\begin{array}{c} \text{Attention}\left(\text{Q},\text{K},\text{V}\right)=\text{softmax}\left(\frac{\text{Q}{\text{K}}^{\text{T}}}{\sqrt{{\text{d}}_{\text{k}}}}\right)\text{V}, \end{array}$$

where *d*_*k*_ denotes the number of dimensions of Q and K.

Meanwhile, multiple scaled dot-product attention will be calculated parallelly in multi-head attention as follows:

(8) $$\begin{array}{c} \text{MultiHead}\left(\text{Q},\text{K},\text{V}\right)=\text{Concat}\left({\text{head}}_{1},{\text{head}}_{2}\cdots {\text{head}}_{\text{h}}\right){\text{W}}^{\text{O}}, \end{array}$$

where *he*a*d*_*i*_ = *Attention*(*QW*_*i*_^*Q*^, *KW*_*i*_^*K*^, *VW*_*i*_^*V*^), *h* is the number of parallel scaled dot-product attention, and *W*^*O*^ ∈ *R*^*hd*_*v*_×*d*_*model*_^ is the parameter matrix.

Mask multi-head attention is similar to the multi-head attention but only keeps the current and previous for every input row.

The feed forward network is a fully connected neural network for every position with a ReLU layer, and a linear layer and can be denoted as follows:

(9) $$\begin{array}{c} FFN\left(x\right)=\max\left(0,xW_{1}+b_{1}\right)W_{2}+b_{2}, \end{array}$$

The add and norm layer will normalize the result of the last layer's output and construct a residual block with the last layer.

### 4.5. Temporal Convolutional Network (TCN)

Temporal convolutional network (TCN) [17] implements the convolutional network for time series. TCN has an excellent performance in capturing the long-term dependency relations and local information. It also keeps the advantage of a convolutional network by extracting features with limited parameters. The structure of TCN is shown in Figure 7.

The convolution operation in TCN is based on the following formula:

(10) $$\begin{array}{c} \text{F}\left(\text{s}\right)=\overset{\text{k}-1}{\underset{\text{i}=0}{\sum }}\text{f}\left(\text{i}\right)∙{\text{x}}_{\text{s}-\text{d}*\text{i}}, \end{array}$$

where *F*(*s*) represents the dilated convolution operation *F* on element *s*, *d* is the dilation factor, and *k* is the filter size.

### 4.6. Deep Autoregressive Recurrent Neural Networks (DeepAR)

DeepAR [18] combines recurrent neural networks and the autoregressive model. Instead of a determined value, it will output a probability distribution of the prediction value. Regrading to the feature of autoregressive regression, DeepAR has a better performance on data with noises.

DeepAR can be represented as follows:

(11) $$\begin{array}{c} {\text{Q}}_{\Theta }=\left({\text{z}}_{\text{i},{\text{t}}_{0}:\text{T}}\left|{\text{z}}_{\text{i},1:{\text{t}}_{0}-1,}{\text{x}}_{\text{i},1:\text{T}}\right.\right)=\overset{\text{T}}{\underset{\text{t}={\text{t}}_{0}}{\prod }}{\text{Q}}_{\Theta }\left({\text{z}}_{\text{i},\text{t}}\left|{\text{z}}_{\text{i},1:\text{t}-1,}{\text{x}}_{\text{i},1:\text{T}}\right.\right)=\overset{\text{T}}{\underset{\text{t}={\text{t}}_{0}}{\prod }}\ell \left({\text{z}}_{\text{i},\text{t}}\left|\theta \left({\text{h}}_{\text{i},\text{t}},\Theta \right)\right.\right), \end{array}$$

where *x*_*i*,*t*_ is the current input covariates, *z*_*i*,*t*−1_ denotes the target value of last time step, 1 : *t*_0_ − 1 is the conditional range, and *t*_0_ : *T* represents the prediction range. *h*_*i*,*t*_= h(*h*_*i*,*t*−1,*z*_*i*,*t*−1_,*x*_*i*,*t*_,_Θ) is the output of the autoregressive recurrent network.

The training process and prediction process are separately shown in Figures 8 and 9. The difference between the two figures is that the prediction range data is unknown in the prediction. The model cannot receive the real value of the last time step but estimates the $\;{\tilde{Z}}_{i,t-1}$ from the sample.

## 5. Results

### 5.1. Experiment

The experiment was based on two research hypotheses: (1) The state-of-art time-series deep learning model will have the better performance on predicting the trend of Indian COVID-19 epidemic, and (2) the vaccination data and population mobility data will be helpful for the accuracy of the model.

The dataset was divided into a training dataset, covering from October 1, 2020, to June 30, 2021, and a testing dataset, covering from July 1 to July 15, 2021. As a preprocessing step, the min-max normalization has been implemented in the training process. The models are fit with the training dataset and then evaluated with the testing dataset. For the logistic regression and multiple linear regression, a single model is trained for a single state, with all features as input and the current state's number of confirmed cases as the label. For other models, all the states share a single and common model.

The root mean square error (RMSE) has been used as the evaluation metric, which is calculated as follows:

(12) $$\begin{array}{c} RMSE=\sqrt{\frac{1}{N}\overset{N}{\underset{i=1}{\sum }}{\left(y_{\text{i}}-{\overset{\wedge }{y}}_{\text{i}}\right)}^{2}}, \end{array}$$

where *y*_*i*_ and ${\hat{y}}_{i}$ are observed and predicted value and *N* is the number of data samples in the test set.

In this research, all the models will predict 15-days confirmed number for every state, and the average RMSE value is used as the main performance measure:

(13) $$\begin{array}{c} {RMSE}_{\text{avg}}=\frac{1}{S}\overset{S}{\underset{i=1}{\sum }}{RMSE}_{\text{i}}, \end{array}$$

where *S* in the number of states in the dataset and *RMSE*_*i*_ is the current state's RMSE value.

The machine learning model is implemented with the open-source Python library dart. Another open source Python library called hyperopt was used for hyperparameter optimization with a stochastic search strategy. The optimization was performed for 100 turns for each model, and the optimal hyperparameters were selected.

### 5.2. Result Table

Table 4 shows the result of the experiment. The training time in hours is also recorded and listed in Table 4.

We can see that the Transformer, as the state-of-art algorithm, performed the best among six models. However, the cost is that the Transformer also took the most time in training. LSTM is less accurate than the Transformer but costs much less time. The traditional statistic methods are not effective in predicting the trend of COVID-19.

### 5.3. Feature Selection

Recall that three feature groups have been used in this research, which are Dose, Google mobility, and Facebook mobility. Considering the contribution of three feature groups to the prediction result, three Transformer models are trained with two feature groups for predicting the number of confirmed and deaths daily number of COVID-19. More specific explanation is given in Table 5.

The results have been shown in Table 6 and Table 7.

As shown in Table 6, mobility data are helpful in predicting, and Facebook mobility dataset contributes the most to the model. It is unexpected that the vaccination rate did not have a positive effect on the prediction. It may cause by the limited immune rate in India; up to July 15, about 23% of the population has been vaccinated one dose, and only 5.8% of the whole population are fully vaccinated. Another potential reason is that the Indian vaccination does not show a stable effect for the new variant virus.

According to Table 7, we can find that the dose and mobility features bring limited effect in forecasting the number of daily deaths of COVID-19. Considering the lagging of vaccination effect, the dead may not be vaccinated or fully vaccinated, and the effect may need to be observed in the longer term.

### 5.4. Discussion

According to the experiment, there are two research hypotheses: (1) The Transformer as the state-of-art time-series deep learning model has a significant better performance than other regression and deep learning models and (2) the population mobility data are helpful for the prediction of spread of epidemic. However, the vaccination data did not have positive effect in predicting.

For the transmission of novel coronavirus, the effect of vaccination is still under the question. Considering the potential variation of the virus, the government should not overlay rely on the vaccination. Meanwhile, the population mobility is an important factor for controlling the spread of epidemic.

## 6. Conclusion

In this study, the COVID-19 epidemic in India was analyzed using datasets collected from different sources. Among the various machine learning models for predicting COVID-19 transmission, the Transformer proved to have the best performance. The Transformer model may be a new baseline for future researchers. The Facebook mobile dataset was found to be most useful along with other datasets in predicting the number of confirmed cases, but not as useful in predicting the number of deaths.

Although the focus area of our study is India, our analysis process can be extended to other countries and regions as long as the original dataset can be collected and used. Another research direction is to find out about COVID-19 between different countries, which may interact with each other.

## Figures and Tables

**Figure 1:** The COVID-19 India dataset read in CSV format.

**Figure 2:** The sample of MoHFW Vaccination data.

**Figure 3:** Procedure of data preprocessing.

**Figure 4:** The structure of a typical LSTM cell.

**Figure 5:** (LSTM) neural networks; *L* represents the cell of Figure 4.

**Figure 6:** The architecture of Transformer.

**Figure 7:** The architecture of TCN.

**Figure 8:** The training process of DeepAR. L is the cell of LSTM.

**Figure 9:** The prediction process of DeepAR.

**Table 1:** Raw data sources.

Raw data sources
COVID-19 India^a^
MoHFW Vaccination^b^
Indian census 2011
Google mobility [9]
Facebook mobility [10]

^a^Data source website: http://www.covid19india.org/. ^b^Ministry of Health and Family Welfare: https://www.mohfw.gov.in/.

**Table 2:** Raw dataset description.

Raw data sources		
COVID-19 India	Level	State
	Storage format	Json/csv

MoHFW Vaccination	Level	State
	Storage format	PDF

Indian census 2011	Level	District
	Storage format	Website
	Variable	Description
	District	The name of district
	State	The state which the district belongs to
	Population	The population number of the district
	Growth	The growth of population number since last census
	Sex ration	The ratio of number of male and female
	Literacy	The percentage of literacy in the state

Google mobility	Level	State
	Storage format	CSV
	Variable	Description
	Grocery and pharmacy	Mobility trends for places like grocery markets
	Parks	Mobility trends for parks
	Transit stations	Mobility trends for public transport hubs
	Retail and recreation	Mobility trends for retail and recreation
	Residential	Mobility trends for places of residence
	Workplaces	Mobility trends for places of work

Facebook mobility	Level	District
	Storage format	CSV
	Variable	Description
	all_day_bing_tiles_visited_relative_change	Positive or negative change in movement relative to baseline
	all_day_ratio_single_tile_users	Positive proportion of users staying put within a single location

**Table 3:** Feature explained.

Variable	Description
dateymd	The date of tuple of data
confirmed	The number of daily confirmed
recovered	The number of daily recovered
deaths	The number of daily deaths
Dose1	The cumulative ratio of population injected first vaccination
Dose2	The cumulative ratio of population injected second vaccination
Grocery & pharmacy	Mobility trends for places like grocery markets
Parks	Mobility trends for parks
Transit stations	Mobility trends for public transport hubs
Retail & recreation	Mobility trends for retail and recreation
Residential	Mobility trends for places of residence
Workplaces	Mobility trends for places of work
visit	Positive or negative change in movement relative to baseline
staying	Positive proportion of users staying put within a single location

**Table 4:** Results of different models.

Model	*RMSE*_*avg*_	Training time (hours)
LSTM	584.74	2.33
Transformer	460.08	11.1
Logistic regression	971.89	0.03
Multiple linear regression	1885.12	0.01
TCN	1605.52	1.12
DeepAR	927.79	4.36

**Table 5:** The explanation of feature selection models.

Model	Description
Baseline (Transformer)	The transformer model training with all features
Transformer_without_dose	The transformer model training without dose feature group, which are Dose1 and Dose2 as shown in Table 3
Transformer_without_google	The transformer model training without Google mobility feature group, which are grocery and pharmacy parks, transit stations, retail and recreation, residential, and workplaces as shown in Table 3
Transformer_without_facebook	The transformer model training without Facebook mobility feature group, which are visit and staying as shown in Table 3

**Table 6:** Transformer model with feature selection for predicting the number of confirmed cases.

Transformer model with feature selection (confirm)	
Model	*RMSE*_*avg*_
Baseline (transformer)	460.08
Transformer_without_dose	426.47
Transformer_without_google	519.28
Transformer_without_facebook	1105.17

**Table 7:** Transformer model with feature selection for predicting the number of deaths.

Transformer_deaths model with feature selection	
Model	RMSE
Baseline (transformer)	103.80
Transformer_without_dose	31.22
Transformer_without_google	45.09
Transformer_without_facebook	26.89

## Data Availability

The datasets used and/or analyzed during the current study are available from the corresponding author on reasonable request.
